RETRACTED

# Changes of Mental State and Serum Prolactin Levels in Patients with Schizophrenia and Depression after Receiving the Combination Therapy of Amisulpride and Chloroprothixol Tablets

**DOI:** 10.1155/2022/6580030

**Published:** 2022-02-22

**Authors:** Bozhi Yuan, Mei Yuan

**Affiliations:** Department of Psychiatry, Hanyang Hospital Affiliated to Wuhan University of Science and Technology, Wuhan 430051, China

## Abstract

**Objective:**

To investigate the changes in mental state and serum prolactin levels in patients with schizophrenia and depression after receiving the combination therapy of amisulpride and chloroprothixol tablets.

**Methods:**

A total of 148 schizophrenic patients with depression were randomly divided into control group (*N* = 73) and study group (*N* = 75). The control group was treated with clopidothiol, and the study group was treated with amisulpride. Symptom scores, sleep quality, adverse reactions, therapeutic effects, prolactin, and progesterone levels, HAMD, PANSS, and PSP scores were compared between the two groups.

**Results:**

The symptom scores of both groups were significantly reduced, but when compared to the control group, the symptom scores of the research group were significantly reduced more significantly (*P* < 0.05); serum GDNF levels of both groups were significantly increased, while serum NSE, IL-1, and MBP levels were significantly reduced (*P* < 0.05). However, the research group altered more substantially (*P* < 0.05) than the control group; the overall PSQI score of the research group was lower (*P* < 0.05) than the control group; and the incidence of adverse responses in the control and study groups was 12.3 percent and 4.0 percent. The research group had a lower rate of adverse responses (*P* < 0.05) than the control group, and the effective treatment of the control and research groups was 82.2 percent and 98.7%, respectively. The research group had a lower rate of adverse reactions (*P* < 0.05) than the control group, while the control and research groups' successful treatment rates were 82.2 percent and 98.7%, respectively. When compared to the control group, the research group had a greater treatment efficiency (*P* < 0.05); blood prolactin and progesterone levels were considerably lowered in both groups, but the reductions in the research group were more evident (*P* < 0.05). Both groups had considerably lower HAMD and PANSS scores, and both had significantly higher PSP scores, although the difference in the research group was more evident (*P* < 0.05).

**Conclusion:**

For people with schizophrenia and depression, a combination of amisulpride and chloroprothixol pills has a considerable effect. It can help patients with their clinical symptoms and sleep quality while also lowering their serum prolactin levels, which is favorable to their illness recovery. As a result, the combined treatment of amisulpride and chloroprothixol pills deserves to be promoted and used.

RETRACTED

## 1. Preface

People's lives are now more stressful than they have ever been, and the frequency of schizophrenic groups is increasing year after year. Some patients may have depressive symptoms, which will disrupt their normal sleep patterns and have a greater effect on their overall quality of life [1]. Drugs are often used in clinical adjuvant treatment, however, patients frequently have serious pharmaceutical adverse effects. In therapeutic settings, chloprothixol tablets are used to treat people with schizophrenia and depression. However, prolactin secretion will be altered to some degree following pharmaceutical treatment, and patient compliance will be limited [2]. Due to sensitivity to adverse responses, some patients may stop taking the treatment or lower their dosage, resulting in recurrent illnesses that are difficult to manage [3]. Amisulpride therapy is based on the use of Chloprothixol pills, which have a good therapeutic effect and are quite safe. It is an atypical antipsychotic medication that is a benzamide derivative [4].

A total of 148 individuals with schizophrenia and depression were chosen for this trial, and they were given amisulpride and chloroprothixol pills. The research looked at changes in patients' mental states and serum prolactin levels in the hopes of improving the patients' mental health and prognosis, as well as the treatment's safety.

## 2. Materials and Methods

### 2.1. The General Materials

The control group (*n* = 73), 35 males and 38 females, with an average course of disease (5.60.6) years, age 18-60 years old, average age (32.42.6) years old; the research group (*n* = 75), 36 males and 39 females, average course of disease (5.50.6) years, age 18-60 years old, average age (32.62.4) years old; the research group (*n* = 75), 36 males and 39 females, average course of disease (5.50.6) years, age 18-60 criteria for inclusion [5]: (1) did not take part in any other clinical trials during the research; (2) age ≥ 18 years old; (3) obvious clinical symptoms, diagnosed as schizophrenia with depression after diagnosis; (4) cooperate with the study and be able to receive prognostic follow-up; (5) first onset. Exclusion criteria: (1) intolerance to the study drug; (2) breastfeeding or pregnancy; (3) with coronary heart disease, hyperthyroidism, and other physical diseases; (4) having a suicidal tendency; (5) receiving antipsychotic medication 12 months before admission. The research subjects agreed with the study, the data were comparable (*P* > 0.05), and the hospital ethics committee agreed.

RETRACTED

### 2.2. Method

Amisulpride is a drug that is used to treat a variety (National Medicine Standard H20113231, manufacturer: Qilu Pharmaceutical Co., Ltd.) treatment: 1000 mg/time, 1 time per day; the first week's treatment is continued at a daily dose of 300 mg. This dose should be continued if the patient has no visible adverse events; the patient had a total of 12 rounds of continuous treatment. Chloprothixol tablets (National Medicine Standard H31021424, manufacturer: Shanghai Xinyi Pharmaceutical Co., Ltd.) treatment: 1 time/day, 5 mg/time, gradually increase the dosage after 14 days of treatment, 15-20 mg per day, the patient received a total of 12 courses of continuous treatment.

### 2.3. The Observation Index

The symptom score: record the negative symptoms score, positive symptoms score, and total score, the lower the score is, the more obvious the improvement of symptoms is.

The sleep quality [6]: the Pittsburgh Sleep Quality Index (PSQI) scale is used to assess the patients' sleep quality. The scale includes a total score of 21 points and seven components, each of which has a value of 0-3. The lower the score, the more noticeable the sleep quality improvement is.

The levels of serum GDNF, NSE, IL-1*β*, and MBP [7]: 3 ml fasting venous blood is drawn, centrifuged at a speed of 3000 revolutions per minute, and detected by an automatic microplate reader.

The levels of myelin basic protein (MBP), glial-derived neurotrophic factor (GDNF), neuron-specific enolase (NSE), and interleukin-1*β* (IL-1*β*), relevant operations are carried out in accordance with the instructions. Shanghai Xuya Biotechnology Co., Ltd. provides the kits.

The adverse reactions: count the number of cases of constipation/dry mouth, abnormal liver function, and extrapyramidal reactions, and calculate the incidence.

The following is the therapeutic impact [8]: ineffective: after therapy, clinical symptoms do not improve or deteriorate significantly. Effective: after therapy, the number of patients with positive symptoms drops considerably, and clinical symptoms improve. Significantly effective: clinical problems largely subside after therapy, and mental state noticeably improves. The effective rate is derived by multiplying the total number of cases by 100 percent and adding the number of strikingly effective and effective instances. Prolactin and progesterone concentrations [9]: an electrochemiluminescence immunoassay analyzer is used to test prolactin and progesterone levels. The stronger the therapeutic impact, the more the numbers tend to be normal.

RETRACTED

The HAMD, PANSS, and PSP scores [10]: the depression status of patients was evaluated by the Hamilton Depression Scale (HAMD), and the corresponding scores for severe, moderate, mild depression, and normal were >35 points, 20-35 points, 8-20 points, and <8 points, respectively, the lower the score is, the lighter the depression is. The degree of psychosis symptoms is analyzed through the PANSS scale, including the general psychosis scale, negative symptom scale, and positive symptom scale. Each scale corresponds to 16 items, 7 items, and 7 items. The lower the score is, the lighter the depressive symptoms are. The PSP scale is used to evaluate a personal social function, including self-care, social relations, work, and study. The higher the score is, the more obvious the improvement of social function is.

### 2.4. The Statistical Methods

After that, the data was put through a normal distribution test. The composition ratio should characterize the count data if the data has a normal distribution, and the differences between groups were explored using the chi-square test [11–13]. The measurement data should be expressed as (mean standard deviation), the *t* test should be used to examine the differences between groups, and the physical influencing factors of the case group should be investigated using Logistic regression *P*0.05 is considered statistically significant. GraphPad Prism 8 was used in this study to create graphs.

## 3. Result

### 3.1. The Comparison of Symptom Scores between the Two Groups before and after Treatment

Before treatment, there was no significant difference in the negative, positive, and total symptom scores between the two groups (*P* > 0.05). After treatment, the symptom scores of the two groups were significantly reduced, but compared with the control group, the symptom scores of the research group were reduced more obviously, the difference between the two groups was statistically significant (*P* < 0.05) (Tables 1–3).

### 3.2. The Comparison of the Adverse Reaction Rates between the Two Groups

The adverse reaction rates of the control group and the research group were 12.3% and 4.0%, respectively. Compared with the control group, the adverse reaction rate of the research group was lower. The difference between the two groups was statistically significant (*P* < 0.05) (Figure 1).

### 3.3. The Comparison of the Treatment Effect between the Two Groups

The treatment effect of the control group and the research group was 82.2% and 98.7%, respectively. Compared with the control group, the research group had a higher treatment efficiency. There was a statistically significant difference between the two groups (*P* < 0.05) (Figure 2).

RETRACTED

### 3.4. The Comparison of the Levels of Prolactin and Progesterone in the Two Groups

There was no significant change in prolactin and progesterone levels between the two groups before treatment (*P* > 0.05). The levels of blood prolactin and progesterone in both groups were considerably lowered after treatment, but the changes in the research group were more significant than the changes in the control group, and the difference between the two groups was statistically significant (*P*0.05) Figures 3(a) and 3(b).

### 3.5. The Comparison of the HAMD, PANSS, and PSP Scores of the Two Groups

Before treatment, the HAMD, PANSS, and PSP scores of the two groups were not significantly different (*P* > 0.05). After treatment, the HAMD and PANSS scores of the two groups were both significantly reduced, and the PSP scores were significantly increased, but the changes in the research group were more obvious, and the difference between the two groups was statistically significant (*P* < 0.05) (Figure 4).

### 3.6. The Serum Levels Were Compared between the Two Groups before and after Treatment

Before treatment, there was no significant difference in the levels of serum GDNF, NSE, IL-1*β*, and MBP between the two groups (*P* > 0.05). After treatment, the levels of serum GDNF were significantly increased, and serum NSE, IL-1*β*, and MBP were significantly reduced, but compared with the control group, the changes in the research group were more obvious, and the difference between the two groups was statistically significant (*P* < 0.05) (Table 2).

### 3.7. The Comparison of Sleep Quality Scores between the Two Groups

Compared with the control group, the total PSQI score of the research group was lower, and the difference between the two groups was statistically significant (*P* < 0.05) (Table 3).

### 3.8. The Comparison of the Adverse Reaction Rates between the Two Groups

The adverse reaction rates of the control group and the research group were 12.3% and 4.0%, respectively. Compared with the control group, the adverse reaction rate of the research group was lower. The difference between the two groups was statistically significant (*P* < 0.05) (Figure 1).

### 3.9. The Comparison of the Treatment Effect between the Two Groups

The treatment effect of the control group and the research group was 82.2% and 98.7%, respectively. Compared with the control group, the research group had a higher treatment efficiency. There was a statistically significant difference between the two groups (*P* < 0.05) (Figure 2).

### 3.10. The Comparison of the Levels of Prolactin and Progesterone in the Two Groups

Before treatment, there was no significant difference in the levels of prolactin and progesterone between the two groups (*P* > 0.05). The levels of blood prolactin and progesterone in both groups were considerably lowered after treatment, but the changes in the research group were more significant than the changes in the control group, and the difference between the two groups was statistically significant (*P* > 0.05) (Figures 3(a) and 3(b)).

RETRACTED

### 3.11. The Comparison of the HAMD, PANSS, and PSP Scores of the Two Groups

Before treatment, the HAMD, PANSS, and PSP scores of the two groups were not significantly different (*P* > 0.05). Both groups' HAMD and PANSS scores were considerably reduced after treatment, while their PSP scores were significantly increased, although the changes in the research group were more noticeable, and the difference between the two groups was statistically significant (*P* < 0.05) (Figure 4).

## 4. Discussion

Schizophrenia is caused by a variety of reasons, the most common of which is a loss of serotonin system function. It is also linked to psychotic symptoms and secondary causes. Other psychosocial variables and antipsychotic medications are also linked to it [14–16]. Schizophrenia patients may exhibit both negative and positive symptoms [17]. Hypovolemia, social withdrawal, poor thinking, sluggish movement, lethargy, and other negative symptoms are the most common, whereas thinking disorder, abnormal hyperactivity, hallucinations, uncoordinated actions, delusions, and other positive symptoms are the most common [18]. There are a lot of research on clinical symptoms in the clinical application of amisulpride, however, there aren't enough studies on sleep and mental state improvement. This research examines the safety of the amisulpride therapy by selecting certified samples [19–21]. The findings showed that amisulpride medication for schizophrenia and depression patients has a substantial impact and may help with sleep problems. Because of its evident pharmacological properties, it may help patients' mental states improve even more, and their negative feelings can be greatly reduced [22, 23].

Amisulpride has an antagonistic impact on the midbrain-limbic system's postsynaptic membrane dopamine receptors. The primary considerations are the pharmacological properties. The release and synthesis of dopamine are greatly enhanced, and the transmission speed of dopamine is accelerated. Increasing the quantity of amisulpride prevents the binding between postsynaptic membrane receptors and dopamine and subsequently antagonizes dopamine autoreceptors. The impact of amisulpride on 5-HT7a is now causing a lot of clinical worry. Some researchers think it is linked to the antidepressant effect. Patients with positive and negative symptoms are visible, and some patients will have significant cognitive impairment, act oddly, and be prone to crankiness. A combination of amisulpride and chloroprothixol tablets therapy, according to some experts, has a greater impact.

RETRACTED

The brain's postsynaptic dopamine receptors are blocked by chlorprothixol tablets. It is an antipsychotic that may assist with depression and anxiety [22]. The research looked at the impact of combining two medications on patients' mental health and clinical symptoms. The study's findings revealed that both groups' symptom scores were significantly reduced, but the research group's symptom scores decreased more significantly (*P* < 0.05) when compared to the control group; both groups' HAMD and PANSS scores were significantly reduced, and both groups' PSP scores were significantly increased, but the changes in the research group were more significant (*P* < 0.05). The findings revealed that, when compared to single-drug treatment, two-drug combination therapy may significantly improve clinical symptoms while also alleviating depression in patients. Patients' ability to communicate emotions and sleep quality may both be enhanced. Patients with schizophrenia and depression have apparent nervous system impairment, and their serum MBP and NSE levels will be much higher. Clinical monitoring of GDNF levels may be used to assess a patient's cognitive function. Furthermore, some researchers asserted that there is a link between blood IL-1 levels and patient cognitive performance, and that serum IL-1 levels may be used to assess central nervous system degeneration and injury [23]. The study's findings revealed that both groups' serum GDNF levels were considerably higher, while their serum NSE, IL-1, and MBP levels were significantly lower, although the research group altered more significantly (*P* < 0.05) than the control group. The results confirmed that the combined treatment of amisulpride and chloroprothixol tablets is beneficial to the improvement of the central nervous system function of patients, and at the same time reduces the level of serum inflammatory factors, which can speed up the recovery of patients. The combined therapy of amisulpride and chloroprothixol tablets is safer and can improve patients' clinical symptoms. However, clinical attention should be paid to the effect of the above two drugs on the serum prolactin level of patients. Under the action of prolactin release inhibitors and prolactin release factors, the amount of prolactin secreted increased significantly [24]. Amisulpride blocks presynaptic autoreceptors, resulting in a considerable improvement in patients' unpleasant feelings. According to the findings, the incidence of adverse responses in the control and research groups was 12.3 percent and 4.0 percent, respectively, and the successful treatment rate was 82.2 percent and 98.7%, respectively. In comparison to the control group, the research group had a higher treatment efficiency and a lower incidence of adverse reactions (*P* < 0.05); both groups had substantial decreases in blood prolactin and progesterone, albeit the reductions in the research group were more significant (*P*0.05) when compared to the control group. When compared to single-drug therapy, the data showed that combining the two medicines may enhance blood prolactin and progesterone levels to a greater degree while also improving patient prognosis and treatment compliance. To conclude, the combined therapy of amisulpride and chloroprothixol tablets for schizophrenia and depression improves clinical symptoms and sleep quality while reducing serum prolactin levels, which is beneficial to recovery. As a result, the combination therapy of amisulpride and chloroprothixol pills deserves to be promoted and used.

RETRACTED

## Figures and Tables

**Figure 1:** The comparison of the adverse reaction rates between the two groups.

**Figure 2:** The comparison of the treatment effect between the two groups.

**Figure 3:** The comparison of the levels of prolactin and progesterone.

**Figure 4:** The comparison of the HAMD, PANSS, and PSP scores of the two groups.

**Table 1:** The comparison of the symptom scores between the two groups before and after treatment ($\bar{x}\pm s$).

Group	Number of cases	The negative symptom score		The positive symptom score		Total score	
		Before treatment	After treatment	Before treatment	After treatment	Before treatment	After treatment
The control group	73	27.6 ± 1.9	20.5 ± 1.5	14.2 ± 2.6	8.6 ± 1.5	80.7 ± 3.8	66.5 ± 3.2
The research group	75	27.5 ± 2.0	18.2 ± 1.3	13.8 ± 2.4	7.8 ± 1.8	80.6 ± 3.7	50.8 ± 2.7
*T*	/	1.526	15.724	0.963	13.728	0.514	18.725
*P*	/	>0.05	<0.05	>0.05	<0.05	>0.05	<0.05

**Table 2:** The comparison of the serum levels between the two groups before and after treatment ($\bar{x}\pm s$).

Group	Number of cases	GDNF (pg.mL^−1^)		NSE (*μ*g. L^−1^)		IL-1*β* (*μ*g. L^−1^)		MBP (*μ*g. L^−1^)	
		Before treatment	After treatment	Before treatment	After treatment	Before treatment	After treatment	Before treatment	After treatment
The control group	73	354.9 ± 38.6	522.5 ± 57.3	33.4 ± 4.6	22.7 ± 3.6	51.6 ± 6.5	26.3 ± 4.2	2.8 ± 0.5	2.4 ± 0.4
The research group	75	355.2 ± 38.5	592.33 ± 62.5	33.2 ± 4.5	14.3 ± 2.3	51.8 ± 6.7	18.3 ± 2.6	2.8 ± 0.6	2.0 ± 0.3
*T*	/	1.527	17.628	0.158	15.034	1.985	16.5428	0.854	14.936
*P*	/	>0.05	<0.05	>0.05	<0.05	>0.05	<0.05	>0.05	<0.05

RETRACTED

**Table 3:** The comparison of the sleep quality scores between the two groups ($\bar{x}\pm s$).

Group	Number of cases	Daytime dysfunction	Sleep quality	Sleep disturbance	Sleep time	Sleep efficiency	Time to fall asleep	Total PSQI score
The control group	73	1.7 ± 0.5	1.9 ± 0.7	1.2 ± 0.3	1.5 ± 0.4	1.7 ± 0.6	1.2 ± 0.7	9.2 ± 3.2
The research group	75	1.3 ± 0.4	1.5 ± 0.4	0.7 ± 0.4	0.9 ± 0.3	1.3 ± 0.5	0.8 ± 0.5	6.5 ± 2.5
*T*	/	0.524	13.854	0.854	13.025	0.421	14.5211	18.325
*P*	/	<0.05	<0.05	<0.05	<0.05	<0.05	<0.05	<0.05

## Data Availability

The data used to support the findings of this study are included within the article.
